The article "Detecting and Extracting Brain Hemorrhages from CT Images Using Generative Convolutional Imaging Scheme" was retracted in 2023. Reasons: signs of a paper mill; compromised peer review; unreliable results or conclusions.

# Detecting and Extracting Brain Hemorrhages from CT Images Using Generative Convolutional Imaging Scheme

**DOI:** 10.1155/2022/6671234

**Published:** 2022-05-06

**Authors:** V. Pandimurugan, S. Rajasoundaran, Sidheswar Routray, A. V. Prabu, Hashem Alyami, Abdullah Alharbi, Sultan Ahmad

**Affiliations:** ^1^School of Computing Science and Engineering, VIT Bhopal University, Madhya Pradesh, India; ^2^Department of Computer Science and Engineering, School of Engineering, Indrashil University, Rajpur, Mehsana, Gujarat, India; ^3^Department of Electronics and Communication Engineering, Koneru Lakshmaiah Education Foundation, Guntur, India; ^4^Department of Computer Science, College of Computers and Information Technology, Taif University, P.O. Box 11099, Taif 21944, Saudi Arabia; ^5^Department of Information Technology, College of Computers and Information Technology, Taif University, P.O. Box 11099, Taif 21944, Saudi Arabia; ^6^Department of Computer Science, College of Computer Engineering and Sciences, Prince Sattam Bin Abdulaziz University, Alkharj 11942, Saudi Arabia

## Abstract

**Purpose:**

The need for computerized medical assistance for accurate detection of brain hemorrhage from Computer Tomography (CT) images is more mandatory than conventional clinical tests. Recent technologies and advanced computerized algorithms follow Artificial Intelligence (AI), Machine Learning (ML), and Deep Learning (DL) techniques to improve medical diagnosis platforms. This technology is making the diagnosis practice of brain issues easier for medical practitioners to analyze and identify diseases with an assured degree of precision and performance.

**Methods:**

As the existing CT image analysis models use standard procedures to detect hemorrhages, the need for DL-based data analysis is essential to provide more accurate results. Generally, the existing techniques are limited with image training efficiency, image filtering procedures, and runtime system tuning modules. On the scope, this work develops a DL-based automated analysis of CT scan slices to find various levels of brain hemorrhages. Notably, this proposed system integrates Convolutional Neural Network (CNN) and Generative Adversarial Network (GAN) architectures as Integrated Generative Adversarial-Convolutional Imaging Model (IGACM) for extracting the CT image features for detecting brain hemorrhages.

**Results:**

This system produces good results and takes lesser training time than existing techniques. This proposed system effectively works over CT images and classifies the abnormalities with more accuracy than current techniques. The experiments and results deliver the optimal detection of hemorrhages with better accuracy. It shows that the proposed system works with 5% to 10% of the better performance compared to other diagnostic techniques.

The article "Detecting and Extracting Brain Hemorrhages from CT Images Using Generative Convolutional Imaging Scheme" was retracted in 2023. Reasons: signs of a paper mill; compromised peer review; unreliable results or conclusions.

**Conclusion:**

The complex nature of CT images leads to noncorrelated feature complexities in diagnosis models. Considering the issue, the proposed system used GAN-based effective sampling techniques for enriching complex image samples into CNN training phases. This concludes the effective contribution of the proposed IGACM technique for detecting brain hemorrhages than the existing diagnosis models.

## 1. Introduction

The main causes of brain hemorrhage are blood pressure, consumption of alcohol, and heredity. A patient's response to a brain hemorrhage depends on the size of the hemorrhage and the amount of distension. The hemorrhage is divided into different categories using the CT images. They are mentioned as Intraventricular Hemorrhage (IVH), Intracerebral Hemorrhage (ICH), Subarachnoid hemorrhage (SAH), Epidural hemorrhage (EDH), and Subdural hemorrhage (SDH) [1, 2].  Figure 1 illustrates the different types of brain hemorrhages in detail [Pinterest Medical portal].

The existing CT image analysis techniques and other clinical practices have low sensitivity to detecting minor nonhemorrhagic issues. Analyzing the CT image features using linear and nonlinear classification models is more useful to deliver flawless results. Under most of the cases, CT images are scanned using bottom to top fashion that moderates the quality of nasal cavity slices. This degrades the successful detection of abnormal issues of the brain. Generally, CT is the optical imaging procedure used for detecting severe head trauma, and it allows for precise diagnosis assistance [3]. Compared to other scanning methods, CT scanning tools provide fast image acquisition time, early symptoms of a brain hemorrhage. In this regard, this CT imaging technology is preferred over other tools. CT imaging technique uses X-ray beams to create a sequence of brain photographs, where the brain tissues are filled with varying intensities based on the tissue's X-ray absorbency.

Currently, several models are used to diagnose brain hemorrhage, bone fractures, and tumors. However, the deep extraction and suitable training models make crucial impacts on the extraction of CT image features to detect brain hemorrhages. The existing systems use either conventional clinical approaches or computerized decision-making systems. Compared to generic clinical techniques, ML- and DL-based computerized techniques are more effective [4, 5]. In this regard, many CT image analysis models implemented ML-based classification techniques and DL-based techniques such as Decision Trees (DT), Support Vector Machine (SVM), CNN, Recurrent Neural Network (RNN), and Boltzmann machines (BM).

The article "Detecting and Extracting Brain Hemorrhages from CT Images Using Generative Convolutional Imaging Scheme" was retracted in 2023. Reasons: signs of a paper mill; compromised peer review; unreliable results or conclusions.

The existing systems developed hemorrhage detection techniques with the help of limited sample generation principles and restricted training models [6–8]. Similarly, they contributed to detecting explicitly located symptoms and image abnormalities for ensuring brain hemorrhages. These efforts are not suitable for the early-stage detection and deep feature extractions of hemorrhage patterns.

To solve these issues, the proposed IGACM implements CNN for effective feature extractions and GAN for finding early state hemorrhage dimensions [9]. This proposed DL-based IGACM develops deep learning structures and diagnostic procedures that can distinguish and detect all of the crucial points from CT images. Secondly, this system assists medical practitioners, clinicians, and doctors in providing accurate therapies. The proposed IGACM is an automated CT image feature classification system that analyzes various CT image slices to detect and differentiate brain hemorrhages. Generally, the existing brain hemorrhage detection techniques were not developed for deeply analyzing the medical image contents. Additionally, the present techniques were focused on MRI data features only. This leads to inaccuracy and increasing diagnosis cost comparing to CT image extraction procedures. This is considered as crucial research problem. On the scope, the proposed system is motivated to implement deeply trained IGACM for diagnosing the CT images of brain hemorrhages for achieving more accuracy. In addition, the proposed IGACM has been motivated to use CT images rather than MRI data to reduce the medical expenses.

In this article, Section 2 presents the materials and methods that describe various related works used for the research study and explain the technical components and working principles of the proposed system.  Section 3 elaborates on the experiments and results obtained.  Section 4 concludes the proposed article with several forthcoming ideas.

## 2. Materials and Methods

Recently developed optical and clinical imaging techniques aid doctors in tracking and saving the patients from a tumor or any abnormal brain tissue growth. Liu et al. [10] suggested a symmetric detection method to identify brain lesions based on preliminary findings.

According to the assumptions, the work tried to find the various brain hemorrhages based on symmetricity pattern evaluations. However, this work produced a lack of accuracy, and it used less efficient classification phases. Chan et al. [11] adapted midline detection techniques using CT images. Burduja et al. [12] presented a systematic approach for hemorrhage detection based on the CNN for ICH detection using CT images. This technique analyzed hemorrhages from CT scan images through a joint RNN and Long Short Term Memory (LSTM) networks. This LSTM based CT image analysis evaluated various slices of brain images and produced the stream of results in abnormality detection (LSTMDS). However, this technique requires more time for training and produced limited accuracy in the image data evaluation platform.

The article "Detecting and Extracting Brain Hemorrhages from CT Images Using Generative Convolutional Imaging Scheme" was retracted in 2023. Reasons: signs of a paper mill; compromised peer review; unreliable results or conclusions.

Chen et al. [13] provided hemorrhage detection schemes based on IoT smart intelligent systems. This work proposed a smart IoT application that accurately diagnoses brain hemorrhage for patients. Tong et al. [14] presented SVM-based feature detection techniques. This scheme provides only basic ML classification with a limited knowledge base. Shuchi et al. [15] mentioned the important parameters and analyzed the CT image slicing techniques like ML-based Statistical Analysis (MLSA), watershed, and Expectation-Maximization (EM) methods. These techniques were implemented with the average training time for classifying the images. Raja et al. [16] presented DL algorithms for the detection of ICH. The authors proposed a generalized additive model and random forest classifier model for slicing and detecting brain abnormalities. Agata et al. [17] proposed intensity windows and consecutive slicing of the image for the detection of a brain hemorrhage. Additionally, this approach performed primary Region of Interest (ROI) extractions to prepare the data for the analysis. Chithra et al. [18] presented the various image processing techniques for considering the image parameters such as color, texture, size, and shape image sections. The author mentioned the main goal of the image enhancement to provide the nonblurred image for the diagnosis and pretended to use SVM and K Nearest Neighbor (KNN) classifier methods for getting the results.

Kamnitsas et al. [19] suggested an effective computational method to overcome the burden of 3D image data analysis schemes. This scheme segmented various image sections as patches for minimizing data extraction loads. Schmitz et al. [20] presented baseline margin techniques with CNN architectures for detecting brain issues (CNNDS). This scheme tried to maintain an optimal spatial relationship between the different image contents in the training model and computational costs. Peng et al. [21] provided the DL-based brain age prediction model that used weighted structural Magnetic Resonance Imaging (MRI) data and CNN-based classification models. For improving the quality of this DL model, the authors investigated the lightweight data analysis schemes and data regularizing schemes in the diagnosis architectures. Nonetheless, these schemes produced significant error rates.

The article "Detecting and Extracting Brain Hemorrhages from CT Images Using Generative Convolutional Imaging Scheme" was retracted in 2023. Reasons: signs of a paper mill; compromised peer review; unreliable results or conclusions.

The proposed system uses CNN and GAN models to solve the above issues. We have various ML and DL techniques for decision-making systems. However, the integration of CNN and GAN makes a crucial impact to improve disease detection accuracy in the medical field.

Compared to other artificial techniques, CNN is more efficient to analyze image features. Subsequently, CNN uses an adaptive layer and filter for feature classification and extraction under optimal training intervals. At the same time, GAN works more actively on crucial sample generation and adversary point discrimination. Thus, the integration of CNN and GAN improves the detection accuracy of brain hemorrhages using CT images.

### 2.1. Research Problem and Motivation

The medical systems require a well-trained computer model to detect brain disorders [22–25]. The artificial diagnosis models gather CT image features, extract the feature point, classify the image point, and provide accurate determinations. The medical imaging techniques are categorized, such as MRI, CT, X-Rays, Positron Emission tomography (PET), and ultrasound emissions. Based on the data acquired and searched for the currently accessible diagnosis schemes, an appropriate system can detect normal injury and hemorrhages. Many recent medical imaging techniques developed CT image feature extraction practices [26, 27]. Additionally, the existing medical imaging techniques need well-defined computerized decision-making systems. In this regard, ML and DL systems were integrated with medical diagnosis models. These systems assist the doctors in observing the brain tissue problems, hemorrhages, with more accuracy rate. Consequently, this helps them take appropriate treatments to patients to save their lives [28]. Anyhow, the existing ML-based CT feature classification systems lacked accuracy and precision rate. Additionally, these techniques were not optimally working to detect minimal quantities of brain tissue disorders and took more training time. Thus, the proposed system is motivated to develop IGACM based CT image analysis tool. This work effectively gathers and extracts the features of CT images to diagnose brain hemorrhages.

Also, this proposed model distinguishes minor damage and brain hemorrhage to prevent tissue loss or serious impairment [29, 30]. The proposed IGACM technique is an automated CT slice analysis method that assists the medics at emergency times.

### 2.2. Proposed IGACM for Detecting Brain Hemorrhages

CT image is analyzed through segmentation and grayscale evaluation procedures [31]. The segmented CT image is stored in a secondary database. In the first phase of the proposed system, these segmented images are given into CNN layers (ConvNets). CNN functions and ConvNet filters extract the image features effectively. At the same time, the trained CNN layers classify the suspected slices from the segments. On the other hand, GAN generates a crucial set of samples from available sample data using the generator function. Consequently, the differentiator function of GAN finds the unobservable brain damage portions using these effective generator samples. This increases the precision and specification rates of proposed IGACM on selected CT images. The experiments on various CT images deal with preprocessing, segmentation, cluster formation, and content evaluation.

The article "Detecting and Extracting Brain Hemorrhages from CT Images Using Generative Convolutional Imaging Scheme" was retracted in 2023. Reasons: signs of a paper mill; compromised peer review; unreliable results or conclusions.

The proposed IGACM initiates various image analysis processes such as image data preprocessing, noise elimination, segmentation, model training, model tuning, and detecting brain tissue problems in respective slices.  Figure 2 illustrates the details of the proposed IGACM components. In this case, the collected CT images are preprocessed for removing noise contents and other distortions. In the next phase, the CT brain images are segmented into different sectors. At the end of these initial setups, the trained CNN filters extract and classify image block contents into the next level process. At the same time, GAN assists the CNN functions by tuning the classification system with the help of complex sample generation functions.

Finally, GAN tunes the CNN-based CT classification model with the help of image discrimination functions. These GAN functions increase the classification accuracy in need. Thus, the proposed IGACM effectively generates various new samples and tunes itself for improving the accuracy of the CT diagnosis system. The significant phases of the proposed IGACM are given as follows. They are data preprocessing, feature extraction, training, tuning, and classification. In complex systems, the image feature points may not be correlated or linear to each other. To this end, the trained DL-based image diagnosis system helps classify the syndromes easily [32–34]. In this work, the diagnosis of the brain hemorrhage reveals various brain portions of the brain image. Once the features are extracted, CT images are segmented into CNN layers. As CT-scan images are gray-level images, visual inspection of these images gives texture criterion to analyze and distinguish the data points. For that purpose, wavelet and Haralick texture models are applied to analyze the images. This work is focusing on texture analysis first and then intensity plots to compare the CT images based on trained parameters. In this texture analysis, the proposed scheme decomposed the image four times using wavelet transform and then reconstructed the image by using detailed coefficients and based on the difference generated using a texture map. Secondly, the proposed scheme calculates the histogram of image intensity distributions and determines the arithmetic mean and standard deviation to compare the diseased images from the normal image. Thirdly, Haralick model texture descriptors help in classifying diseased images from the normal image [35].

The article "Detecting and Extracting Brain Hemorrhages from CT Images Using Generative Convolutional Imaging Scheme" was retracted in 2023. Reasons: signs of a paper mill; compromised peer review; unreliable results or conclusions.

The CT image features used for the experiment purpose are given as follows. These are entropy, energy, contrast, homogeneity, sum mean, variance, maximum probability, and correlation. The images portions with minimal sum and mean were discarded for training the comparison and classification model. Finally, CNN-GAN units classify the normal and abnormal slices. Thus, a report gives the disease diagnosed along with some prescriptions. The CT image database contains the details of 130 patients for training the models. In several experiments, MRI data is preferred. Compared to MRI data, CT images are more suitable for brain hemorrhage detection. Generally, CT images are observed with the help of X-Rays and MRI details are observed through magnetic fields. In this case, CT is more effective to diagnose the tissue impacts, hemorrhages, and other problems. At the same time, CT images are less expensive compared to MRI. Thus, the proposed system uses CT image feature extraction for the benefit of patients.

The process of designing, testing, and verifying a diagnostic model to forecast the probability of tumor occurrence is known as predictive modeling. In predictive modeling solutions, a variety of methods are used such as machine learning, artificial intelligence, and statistics. The diagnosis and predictive models examine the historical knowledge base to forecast future outcomes. The diagnostic model is built after feature extraction and training data deployment. It is a subset of data analytics that detects the outcomes of CT image computations. Similarly, each model is constructed based on the amount of extremely favorable predictors for determining future decisions. An analytical model is created once the data for a given predictor is acquired. The terms “accuracy” and “error” are frequently used to describe categorization performance. The CNN training and GAN-based tuning functions are given in the following equations and Algorithm 1. Initially, CNN gets the image data as pixels to various features trained to build the classification system [36].

(1) $$\begin{array}{c} I^{px}=\frac{I^{i,j}-I^{mI,mJ}}{i,j}. \end{array}$$

Equation (1) depicts the CT image data as pixel points, *I*^*i*,*j*^ and *I*^*mI*,*mJ*^ as real data and mean data, respectively. The numerator *D*^*i*,*j*^ is used as nominal standard deviation (pixel rate). From equation (1), the image initialization is expressed in terms of pixel measurements with large quantities. This equation shows the correlation between all image quantities and the mean value of each image input. It helps initialize each image into CNN input function with appropriate measurements (pixel value and mean). The number of hidden layers in CNN for extracting the image details is determined based on image components. In this case, the values *i*, *j* state image pixel coordinates. These values are generated with respect to the ConvNet layers, *c*(*l*) at the duration *c*(*t*).

The article "Detecting and Extracting Brain Hemorrhages from CT Images Using Generative Convolutional Imaging Scheme" was retracted in 2023. Reasons: signs of a paper mill; compromised peer review; unreliable results or conclusions.

In this work, this system uses Haar Wavelet Transform Model (HWT). In this method, the image from the original space is transformed to a predefined new space containing spanned orthogonal wavelets, which help in comparison of image data (deviation in coefficients of normal image forms the basis for comparison). The standard equation of HWT is given in equation (2). It is needed for implementing texture-based image segmentation.

(2) $$\begin{array}{c} W\left(t\right)=\left\{\begin{array}{cc} 1, & \forall i\left(0,0.5\right),\\ -1, & \forall i\left(0.5,1\right),\\ 0, & \text{otherwise.} \end{array}\right. \end{array}$$

Equation (2) indicates that the image pixel values *i* can vary from 0 to 1. According to the image pixel quantity evaluation, the pixels are segmented under different textures. Thus, the proposed system uses HWT.

The CT image of brain section is prescribed as *X*(*i*, *j*, *c*(*l*), *c*(*t*)). Similarly, it is expressed as *X*(*i*, *j*, 0, *c*(*t*)) at the end of ConvNet function. Equation (3) shows the CNN observations as *C*(*i*, *j*, *c*(*l*), *c*(*t*)) with *O*^*c*(*t*)^ input weight vector, and Bias_*O*^*c*(*t*)^ as bias in expected output [37, 38].

(3) $$\begin{array}{c} C\left(i,j,c\left(l\right),c\left(t\right)\right)=O^{c\left(t\right)}\cdot X\left(i,j,c\left(l\right),c\left(t\right)\right)+\text{Bias}\_O^{c\left(t\right)}, \end{array}$$

(4) $$\begin{array}{c} C\left(i,j,c\left(l\right),c\left(t\right)\right)=O^{c\left(t\right)}\cdot X\left(i,j,c\left(l\right),c\left(t\right)\right)+\text{Bias}\_O^{c\left(t\right)}\pm O^{c\left(t\right)}\cdot X\left(i,j,c\left(l\right),c\left(t-1\right)\right), \end{array}$$

(5) $$\begin{array}{c} C\_\text{REL}\left(i,j,c\left(l\right),c\left(t\right)\right)=\text{Max}\left\{0,C\left(i,j,c\left(l\right),c\left(t\right)\right)\right\}. \end{array}$$

Equations (4) and (5) show the details of computed image data and ConvNet RELU functions, respectively. Equation (6) gives the normalized CT image outcomes with normalized weight function and as layer associative bias rate.

(6) $$\begin{array}{c} C\_\text{Norm}\left(i,j,c\left(l\right),c\left(t\right)\right)=w\left(t\right)\left(BF\left(C\left(i,j,c\left(l\right),c\left(t\right)\right)\right)\right). \end{array}$$

Equation (7) states the GAN-based CNN tuning function that contains both the sample generator unit and the sample discriminator unit.

(7) $$\begin{array}{c} G\_C\left(i,j,c\left(l\right),c\left(t\right)\right)=\text{Gen}\left(C\_\text{Norm}\right.\left(i,j,c\left(l\right),c\left(t\right)\right)+\text{Disc}\left(\text{Gen}\right.\left(C\_\text{Norm}\right.\left(i,j,c\left(l\right),c\left(t\right)\right). \end{array}$$

In this work, the IGACM detects and predicts the condition of the human brain or bone by an image featuring, but the data extracted from the image features require the classification to give a systematic and graphical representation of all the diagnostic outcomes. Moreover, this model plots the detectable plots and also checks using various libraries that the data is free from all the null values. In this work, the trained CNN model and GAN tuning model are effectively used to detect brain features [39–41]. Consequently, the time is taken for producing the output between 186 milliseconds and 260 milliseconds. Under this situation, the proposed IGACM works with optimal classification accuracy that assists the medical team in diagnosing the patient's issues. The experiment details and CT image observations are given in Section 3.

The article "Detecting and Extracting Brain Hemorrhages from CT Images Using Generative Convolutional Imaging Scheme" was retracted in 2023. Reasons: signs of a paper mill; compromised peer review; unreliable results or conclusions.

## 3. Results and Discussion

As discussed, Figure 1 illustrates the types of brain hemorrhages [42]. The proposed IGACM enhances the CT feature classification accuracy once the images are passed through the initial preprocessing steps. The proposed system uses the CT image dataset as it comprises 2450 images. Among the images, 1250 images are identified with brain hemorrhages with various shapes. The remaining 1200 images are in normal conditions. These data are collected from 130 patients in various age groups between 20 and 65. The patients involved in this experiment have healthy in terms of other diseases. These images are collected from Radiology Society of North America (RSNA) repositories. This dataset is preprocessed for building training sets and test datasets. In the preprocessing phase, both CNN and GAN initiate data reduction procedures and select optimal features under training sets. The test dataset is applied for managing the system tuning process. This test dataset is completely updated with the help of GAN's crucial samples that increase the system's accuracy.

The article "Detecting and Extracting Brain Hemorrhages from CT Images Using Generative Convolutional Imaging Scheme" was retracted in 2023. Reasons: signs of a paper mill; compromised peer review; unreliable results or conclusions.

In this experiment, Weka 3.8 is used for data preprocessing phases (image features). In the next level, MATLAB and Python 3.8 are used for implementing the proposed IGACM. Initially, the raw image dataset (11.48 Mega Bytes) is extracted for gathering image features. The raw dataset features (3.67 Mega Bytes) are given to Weka, and they are preprocessed (1.98 MB).  Figure 3(a) shows the normal brain images (no hemorrhages).  Figure 3(b) gives the clustered points of the normal image (K-Means). This is represented with grayscale quantities. Figures 4 and 5 show the extracted parts of brain hemorrhages.  Figure 4 illustrates the circular shape of ICH that is extracted from IGACM layers. Similarly, Figure 5 shows the affected parts of the brain due to IVH and SAH issues.

These hemorrhages are denoted in the center portion of the brain and cracks in the brain. In the same manner, SDH and EDH portions are extracted as given in Figure 6. Figure 6(a) shows SDH portions (left side stretches near dura) in the brain image. Figure 6(b) shows EDH sections in the CT image clearly.

Figure 7 illustrates the comparison of classification accuracy between the proposed IGACM and the existing systems such as CNN-based Diagnosis System (CNNDS) and LSTM based Diagnosis System (LSTMDS). Figures 7 and 8 provide the details of both existing and proposed solutions. This shows that the proposed IGACM gives better accuracy and specificity rates compared to other works. In this experiment, system accuracy, specificity, precision, and RMSE are taken as evaluation metrics. System accuracy is defined as the number of true detections (either true positive results and true negative results).

System specificity is stated as the number of negative measurements identified from overall test observations. System precision rate is calculated by the ratio between exactly predicted true cases and the overall true predictions. In the same way, RMSE is termed as the standard deviation of system bias rate during the hemorrhage detection process. This is calculated over the precision rate of the proposed system. The proposed system uses both CNN and GAN models for tuning the CNN irregularities. In addition, the test data used by CNN is frequently updated with the help of GAN-associated sample generation functions. This increases accuracy and specificity compared to other techniques. The same benefit of proposed IGACM increases the precision as given in Figure 9. As similar to Figure 9, Figure 10 delivers Root Mean Square Error (RMSE) for CNNDS, LSTMDS, and IGACM techniques. As discussed, the precision and specificity of proposed system increase against training time and number of epochs. This is related to minimal RMSE production of proposed technique.

The article "Detecting and Extracting Brain Hemorrhages from CT Images Using Generative Convolutional Imaging Scheme" was retracted in 2023. Reasons: signs of a paper mill; compromised peer review; unreliable results or conclusions.

Figure 11 gives the observations of sampling rates. The sampling rate can be defined as the number of data samples produced effectively from the overall data. For example, 0.15 rate of samples indicates that 15% of the data are considered as effective samples compared to the overall dataset.

As the number of effective samples increases, the classification accuracy increases to the optimal range. The comparison of effective sampling shows that the proposed GAN associated CNN utilizes more crucial samples than other systems.

As a result, this works better to identify various brain hemorrhages given in Table 1. The proposed model finds preprocessing state samples and GAN based test samples for runtime tuning procedures. This helps increase the sampling rate to (0.35) in 0 to 1 scale measurement. At the same time, the existing systems give only 0.01 to 0.25 of sampling rates. Table 1 lists the classification accuracy of different brain hemorrhages against the increasing number of epochs. The increasing number of epochs states the effective training completion cycles to produce accurate results. Similarly, Table 2 shows the time complexity and space complexity rates of proposed system. In this experiment, the initial overhead affects computation ability as illustrated in Table 2. However, the increasing number of epochs ensures the gradual reduction of time and space complexities. The reduction in complexities happens due to the nature of GAN and CNN accomplishments (increasing learning rate). Also, the reduction in dynamic sampling and dataset overhead impacts the complexity. The size of huge dataset increases system overhead initially. However, the proposed model gradually decreases the computation overhead as the number of epochs increases. The overall system overhead is reduced during effective training phases of CNN and GAN.

Similarly, the other existing techniques such as LSTMDS and CNNDS achieve better results. However, they are not optimal compared to the proposed system. The reason for the better results of the proposed IGACM against existing systems is the integration of GAN and CNN. As discussed earlier, GAN and CNN units work efficiently in terms of new real-time sample productions to improve the system performance than existing techniques [43]. Consequently, LSTMDS and CNNDS can not work better than the proposed IGACM. Thus, the proposed IGACM contributes to developing an efficient brain hemorrhage classification system.

## 4. Conclusion

The proposed IGACM is an automatic CT scan diagnosis scheme that analyzes the brain slices for detecting various hemorrhages. For detecting irregular or nonlinear brain image slices, the proposed IGACM activates CNN and GAN architectures. This system was trained with various complex brain samples and tuned with the help of GAN practices. This helped doctors with more accuracy observe critical brain trauma, which is difficult to distinguish between brain hemorrhage, and brain damage using conventional CT scan studies. The complex nature of CT images leads to noncorrelated feature complexities in diagnosis models. Considering the issue, the proposed system used GAN-based effective sampling techniques for enriching complex image samples into CNN training phases. This proposed work contributed efficient CT image diagnosis models using CNN and GAN systems.

The article "Detecting and Extracting Brain Hemorrhages from CT Images Using Generative Convolutional Imaging Scheme" was retracted in 2023. Reasons: signs of a paper mill; compromised peer review; unreliable results or conclusions.

The proposed system shall be improved with more CT images for finding the solutions to different brain disorders and neural disorders. At the same time, the proposed IGACM is expected to extract both MRI and CT image features. Since the need for CT and MRI technologies in the advanced medical field is increasing, the future adaptations of the proposed work will target better results.

## Figures and Tables

**Figure 1:** Brain hemorrhages.

**Figure 2:** Proposed IGACM functions.

**Figure 3:** CT images. (a) Obtained CT image. (b) K-Means applied and extracted contents (without brain hemorrhages).

**Figure 4:** CT image: (a) intracerebral hemorrhage and (b) extracted contents.

**Figure 5:** IGACM based content extraction for (a) intraventricular and (b) subarachnoid hemorrhages.

**Figure 6:** Extracted CT image contents for showing (a) subdural and (b) epidural hemorrhages.

**Figure 7:** Classification accuracy.

**Figure 8:** Specificity.

**Figure 9:** Precision.

**Figure 10:** RMSE. In this comparison, the proposed work provides 99.5% of precision, specificity, and accuracy rate. In contrast, CNNDS and LSTMDS generate 84.5% to 95% of optimal results, and they are much less than those of the proposed system.

**Figure 11:** Effective sampling rate.

**Algorithm 1:** IGACM on CT Image Analysis.

**Table 1:** Detection accuracy for different types of hemorrhages (%).

Number of epochs	IVH (%)	SAH (%)	EDH (%)	SDH (%)	ICH (%)
30	89.9	88.9	89.3	90.1	90.2
60	90.2	91.2	91.2	91.5	92.2
90	92.3	93.6	93.8	93.4	94.1
120	95.6	96.7	95.7	95.6	95.3
150	98.7	97.9	97.9	97.7	97.9
180	99.6	99.4	99.7	99.3	99.6

**Table 2:** IGACM-time complexity and space complexity.

Number of epochs	Time (seconds)	Space (kB)
30	110.5	90.5
60	109.5	89.5
90	108.7	87.6
120	100.4	79.4
150	98.3	77.1
180	78.2	68.3

## Data Availability

The data used to support the findings of this study are available from the first author upon request (vpcoe84@gmail.com).
